# Preliminary Study of Gastroprotective Effect of *Aloe perryi* and Date Palm Extracts on Pyloric Ligation-Induced Gastric Ulcer in Experimental Rats

**DOI:** 10.1155/2022/9246785

**Published:** 2022-01-24

**Authors:** Naif Al-Gabri, Gehad M. Elnagar, Sultan A. M. Saghir, Amina El-Shaibany, Sultan F. Alnomasy, Ziyad M. Althafar, Nesreen M. I. M. Elkomy, Mahmoud M. Elaasser, Maisa Siddiq Abdoh, Mohammed Yosri

**Affiliations:** ^1^Veterinary Department, Faculty of Agriculture and Veterinary Medicine, Thamar University, Dhamar, Yemen; ^2^Laboratory of Salam Veterinary Group, Buraydah, Al-Qassim, Saudi Arabia; ^3^Biochemistry Department, Faculty of Pharmacy, Zagazig University, Zagazig 44519, Egypt; ^4^Department of Medical Analysis, Princess Aisha Bint Al Hussein College of Nursing and Medical Analysis, Al-Hussein Bin Talal University, Ma'an, Jordan; ^5^Pharmacognosy Department, University of Sana'a, Pharmacy College, Yemen; ^6^Department of Medical Laboratories Sciences, College of Applied Medical Sciences in Al-Quwayiyah, Shaqra University, Al-Quwayiyah, Riyadh, Saudi Arabia; ^7^Department of Pharmacology and Toxicology, Faculty of Pharmacy, Zagazig University, Egypt; ^8^The Regional Center for Mycology and Biotechnology, Al-Azhar University, 11787 Nasr City, Cairo, Egypt; ^9^Department of Medical Laboratory Sciences, Faculty of Applied Medical Sciences, King Abdulaziz University, Jeddah, Saudi Arabia; ^10^Center of Excellence in Genomic Medicine Research, King Abdulaziz University, Jeddah, Saudi Arabia

## Abstract

**Objective:**

The present study was aimed at investigating the possible antiulcer activities of some natural phytochemicals *Aloe perryi* leaf extract (APLE) and flower extract (APFE) in addition to the date palm seed extract (DPSE) and the oily samples of DPSE in a pylorus ligation-induced ulcer model using ranitidine as a standard antiulcer drug.

**Background:**

Peptic ulcer is a prevalent gastrointestinal disorder due to hypersecretion of gastric acid. It affects four million people worldwide, and 2-10% of these ulcers are perforated and cause bleeding. This increases the risk of morbidity and mortality. So we aimed to introduce a primary study alternatively safe method for treating peptic ulcer.

**Materials and Methods:**

Forty-two Wistar Albino rats of either sex were randomly divided into seven groups (6/each). The pylorus ligation was done to induce ulcer in pretreated albino rats. The antiulcer activities of extracts were estimated at different dose levels (250 and 500 mg/kg) using ranitidine as a standard drug (50 mg/kg). Gastric volume, pH, and total and free acidity as well as ulcer index and percentage of ulcer inhibition were measured to elucidate the antiulcerogenic effects. Histological examination of gastric ulcer was also performed. Statistical analysis for the results was done where *P* < 0.05 was considered statistically significant.

**Results:**

Pylorus ligation for 6 h in control rats resulted in gastric ulcer which was indicated by the accumulation of gastric secretion and increased total acidity and decreased pH. The pretreatment of rats with APLE, APFE, and DPSE in addition to the oily samples of DPSE significantly inhibited the ulcers induced by pylorus ligation. These effects were attributed to significant reductions in total and free acidity, ulcer index, and gastric volume while there is a marked decrease in gastric pH (the antisecretory) as well as mucosal strengthening properties of these phytochemicals.

**Conclusion:**

These findings give these extracts the potential to be a promising tool for the management of gastric ulcer after performing further clinical and experimental studies. Our study demonstrated the promising antiulcer activity of extracts and oils in pyloric ligation-induced gastric ulcer. To the best of our knowledge, this is the first study to explore the antiulcer activity of these extracts; however, further investigations may be recommended for full details about this antiulcerogenic capacity.

## 1. Introduction

The peptic ulcer is considered a worldwide chronic disease affecting millions of people and therefore associated with a higher rate of morbidity and mortality [1]. Many factors are contributing to the development of peptic ulcer such as stress, dietary factors, high production of acid, helicobacter Pylori infection, and the use of nonsteroidal anti-inflammatory drugs [2]. Peptic ulcer results in damage of protective mucosal lining of the stomach and duodenum leading to the ulcerogenic process [3].

The treatment of peptic ulcer mainly depended on using remedies that reduce gastric acid secretion such as antacid, but in the last two decades, new drugs are used like an H2 antagonist and proton pump inhibitors. Ranitidine is an H2 receptor antagonist that competes reversibly with histamine for H2 receptor binding on the basolateral membrane of parietal cells thus inhibiting the secretion of gastric acid. It is the most commonly prescribed drug for treating many gastrointestinal disorders such as peptic ulcer and gastroesophageal reflux disease [4]. Ranitidine is a standard antiulcer drug used in many previous studies of gastric ulcer experimentally induced by pyloric ligation in animal models [5–9].

However, the wide use of these antiulcer medications has many drawbacks such as cost, toxicity, drug-drug interactions, and upsetting some cardiac diseases. Therefore, an attention is paid to find more safe and potent nontoxic drugs. Among these new remedies are the herbal drugs due to their lower cost and side effects as well as easy availability [10, 11].

*Aloe perryi* (*Zanzibar* or *Socotrine aloe*) is localized in Socotra in Yemen, an island east of Somalia. It is rich in many active pharmacological compounds like minerals, lectins, vitamins, glycoprotein, alkaloids, amino acids, anthraquinone glycosides, and many essential oils responsible for various medicinal uses of *Aloe perryi* such as anticancer, antibacterial, analgesic, anti-inflammatory, antitumor, antimicrobial, and antiviral activities [12]. Its effect in healing wounds and burns was also reported [13]. Mothana et al. revealed the use of *Aloe perryi* to combat eye and malaria infections and gastrointestinal disorders such as constipation [14].

Date palm (*Phoenix dactylifera*) is considered an important herbal product used in traditional medicines for its potential benefits for health. Egypt is one of the countries that produce date palm [15]. The palm date seed extract is a good source of various important compounds such as saturated and unsaturated fatty acids, phenolic compounds, tocopherols, and sterols which give the extract valuable properties like antiviral, antioxidant, anticancer, antimicrobial, and hypoglycemic ones [16].

Therefore, this study is aimed at introducing a safe medication for treating peptic ulcer versus using the well-established standard antiulcer drug.

## 2. Materials and Methods

### 2.1. Preparation of Plant Extracts

A plant taxonomist in the Department of Botany, Faculty of Science, Sana'a University, Yemen, authenticated both *Aloe perryi* and date palm seeds. Voucher specimens (#4469, 4467) were deposited in the herbarium of the Pharmacognosy Department, Sana'a University.

#### 2.1.1. *Aloe perryi* Extract

The fresh flowers and green leaves of *A. perryi* were collected during the flowering stage in June to July 2019 from the island of Socotra, Yemen.

Both plant parts were dried under shade, powdered coarsely, and stored in an airtight container. The powdered *Aloe perryi* flowers and leaves were 0.5 kg each of them and then were extracted with ethanol (3 × 10 l) at room temperature using a cold maceration procedure. The combined ethanol extract was concentrated under reduced pressure using a rotary evaporator to obtain a thick dark greenish gummy mass for leaves and a reddish brown semisolid extract for the flowers [17].

#### 2.1.2. Date Palm Seed Extract

Date fruits were collected during the last stage of the ripening process in Hadhramaut City, Yemen, 2019. Seeds were isolated from fruits, then soaked in hot water, and washed to remove any adhered date flesh. The seeds were oven dried at 60°C for a day and then roasted and ground using a mechanical grinder to form a powder followed by a sieving process [18].

#### 2.1.3. Preparation of the Oily Samples of the Date Palm Seed Extract

To get yellow colored oil, five hundred grams (500 g) of powdered seed of *Phoenix dactylifera* was extracted exhaustively with 5 l of methanol while to get red colored oil, three hundred grams (300 g) of powdered seed of *Phoenix dactylifera* was extracted exhaustively with 3 l of hexane. The combined filtrates from each one were evaporated by using a rotary evaporator to get the concentrated crude dark brown seed extract; then, oil is leached out from the seed extract where it is separated and purified by filtration.

#### 2.1.4. Transfer to Powder

All stock solution extracts were prepared in dimethyl sulfoxide (DMSO) due to incomplete dissolving in aqueous solution.

### 2.2. Chemicals and Drugs

Ranitidine was obtained from India (Kopran Pharma Ltd., Mumbai). All chemicals or solvents utilized in this study are of analytical grade and supplied from Sigma-Aldrich Chemical Company (St. Louis, MO, USA).

### 2.3. Animals

Forty-two Wistar albino rats weighing 150-200 g of either sex (8-10 weeks of age) were purchased from the Faculty of Veterinary Medicine, Sana'a University, and maintained under standard husbandry conditions (temp 23 ± 2°C, relative humidity 55 ± 10%, and 12-hour light-dark cycle). Animals were fed with standard laboratory food ad libitum during the study period. All experiments were approved by the institutional Ethical Committee, Faculty of Medicine and Health Sciences, Sana'a University (#no.125-10/3/2019#), following the standard guidelines for the use of laboratory animals.

### 2.4. Experimental Design

Albino rats of either sex were randomly divided into seven groups of six animals each as follows:

- Group 1: control group: rats received only distilled water before one hour from pyloric ligation
- Group 2: ranitidine group: rats received ranitidine which is dissolved in distilled water and given in a dose level (50 mg/kg) (p.o.) and served as a standard drug before one hour from pyloric ligation
- Group 3∗: *A. perryi* leaf extract group (APLE): rats received the *Aloe perryi* leaf extract in dose levels of 250 and 500 mg/kg (p.o.) before one hour from pyloric ligation
- Group 4∗: *A. perryi* flower extract group (APFE): rats received the *Aloe perryi* flower extract in dose levels of 250 and 500 mg/kg (p.o.) before one hour from pyloric ligation
- Group 5∗: date palm seed extract group (DPSE): rats received the date palm seed extract in dose levels of 250 and 500 mg/kg (p.o.) before one hour from pyloric ligation
- Group 6∗: yellow oil group: rats received date yellow oil in dose levels of 250 and 500 mg/kg (p.o.) before one hour from pyloric ligation
- Group 7∗: red oil group: rats received date red oil in dose levels of 250 and 500 mg/kg (p.o.) before one hour from pyloric ligation

Asterisks in groups 3, 4, 5, 6, and 7 indicate that animals were divided into two subgroups to receive two dose levels (250 and 500 mg/kg) of different tested extracts.

### 2.5. Induction of Gastric Ulcer by Pyloric Ligation

The ulcer was induced by the pyloric ligation method of Shay [19]. Rats were fasted for 24 h before operation, in individual cages. After 1 h of drug treatment, they were anesthetized with the help of anesthetic ether; the abdomen was opened by a small midline incision below the xiphoid process. Pyloric portion of the stomach was slightly lifted out and ligated, avoiding traction to the pylorus or damage to its blood supply. The stomach was replaced carefully, and the abdominal wall was closed by interrupted sutures. Rats were sacrificed by an over dose of anesthetic ether after four hours of pyloric ligation. The abdomen was opened, the cardiac end of the stomach was dissected out, and the contents were drained into a glass tube.

The volume of the gastric juice was measured and centrifuged at 2000 rpm for 10 min. From the supernatant, aliquots (1 ml of each) were taken for the determination of pH and total and free acidity. Each stomach was examined for lesions in the forestomach portion and indexed according to severity.

### 2.6. The pH Measurement

A pH meter is used for determining pH after diluting 1 ml of gastric juice aliquot with 1 ml of distilled water.

### 2.7. The Total and Free Acidity Determination

1 ml of distilled water was used to dilute 1 ml of gastric juice aliquot and then transferred to a conical flask (50 ml) with the addition of 2 drops of phenolphthalein indicator (Topfer's reagent for the determination of free acidity). 0.01 NaOH was used for titration until a permanent pink color (canary yellow color for free acidity) was resulted; its consumed volume was determined. The total acidity is expressed as mEq/l by calculating according to Reddy et al.'s formula [20].

### 2.8. Macroscopic Evaluation of Gastric Ulcer

A 10x magnifier lens was used to evaluate the ulcers after opening the stomachs along the greater curvature and rinsing them with saline to eliminate any gastric contents or blood clots. For quantification scores, analysis depended on mucosal color, hemorrhages, and superficial and deep ulcer besides perforation which were numbered as follows: 0 = no changes, 1 = mild or focal, 2 = mild to moderate, and 3 = severe [20].

### 2.9. Histological Examination of the Stomach

A portion of the ulcerated stomach was dissected out and fixed in 10% buffered neutral formalin solution; then, tissues were embedded in paraffin, and solid sections were cut at 5 *μ*m by using a LICA microtome and stained with routine hematoxylin and eosin (H&E). The sections were examined under a light microscope and photomicrographs were taken, and lesion scores were compared according to the following semiquantification assay: 0 = normal appearance, 0.5 = mild changes, 1 = moderate changes, 1.5 = severe changes, 2 = over severity, and 3 = diffused [21].

### 2.10. Statistical Analysis

Results were expressed as mean ± SEM. The significance of association between means was assessed by one way-ANOVA, and the group means were evaluated by Dunnett's post hoc test using the SPSS program version 21. *P* < 0.05 was considered statistically significant.

## 3. Results

### 3.1. Antiulcer Activity of DMSO Solution of the *A. perryi* Leaf Extract (APLE) and Ranitidine in Experimental Rats

The treatment of animals with APLE at 250 mg/kg and 500 mg/kg produced significant reductions in total and free acidity and ulcer index while gastric volume was significantly different only on using the high dose of this extract (*P* < 0.01); pH of the gastric juice was increased as compared to the ulcer control group. Ranitidine resulted in more reduction in the gastric parameters (*P* < 0.001) when compared to the control. The ulcer index demonstrated a higher ulcer inhibition with ranitidine therapy (72.1%) when compared with APLE (39.9% and 62.7%) (Table 1/Figure 1).

### 3.2. Antiulcer Activity of DMSO Solution of the *A. perryi* Flower Extract (APFE) and Ranitidine in Experimental Rats

The APFE showed a significant effect on acid parameters and ulcer index in comparison with ulcer control rats. The higher dose of the flower extract (500 mg/kg) showed more superior effect when compared to the lower dose (250 mg/kg). The ulcer inhibition percentage was 52.8% and 71.7% in APFE at doses of 250 and 500 mg/kg, respectively. Ranitidine, the standard drug, exhibited more ulcer inhibition percentage as compared to the flower extract (72.1%) (Table 2/Figure 2).

### 3.3. Antiulcer Activity of DMSO Solution of the Date Palm Seed Extract (DPSE) and Ranitidine in Experimental Rats

The rats pretreated with the date seed extract and ranitidine demonstrated significant (*P* < 0.001) and dose-dependent reduction in acid parameters and ulcer index as compared to the control ones. More ulcer protection was resulted in animals treated with ranitidine (72.1%) when compared with the date seed group (46.9% and 58.6%) (Table 3/Figure 3).

### 3.4. Antiulcer Activity of DMSO Solution of Oily Samples of the Date Palm Seed Extract and Ranitidine in Experimental Rats

Oral administrations of oily samples of the date seed extract either yellow or red demonstrated significant decreases in all estimated acid parameters and ulcer index as compared to the control. The antiulcerogenic effect of yellow or red oil on using dose 500 mg/kg was higher than that on using dose 250 mg/kg. Red oil resulted in more decline in gastric volume and ulcer index as compared to yellow oil at a dose equal to 500 mg/kg. The extracts exhibited gradual protections in ulcer as follows: red oil (82%, 500 mg/kg; 62%, 250 mg/kg) and yellow oil (55%, 500 mg/kg; 32%, 250 mg/kg). Ranitidine showed significant reduction when compared to the control (*P* < 0.001) and resulted in high ulcer inhibition percentage (72.1%) (Table 4/Figure 4).

### 3.5. The Effects of DMSO Solution of the Different Extracts on the Macroscopic Finding of Gastric Ulcer in Experimental Rats

The gross findings in the control group revealed severe ulcer without perforation, while other treatment groups showed mild and moderate to minute ulcer which is noticed to decrease gradually and summarized in Table 5.

### 3.6. The Effects of DMSO Solution of the Different Extracts on the Histological Findings of Gastric Tissue in Experimental Rats

Histological assessment of the gastric mucosa showed that pyloric ligation with the distal water oral group resulted in detachment of mucosal cells, congested blood vessels, and huge submucosal edema with lymphocytic infiltration as an inflammatory aggregate (Figures 5(a)–5(c)). Pretreatment with the different extracts considerably reduced these changes in the gastric mucosa and provided protection against gastric damage (Figures 5(d)–5(f)), besides significantly inhibiting the formation of these lesions' severity and restoring the mucosal damage as summarized in Table 6.

## 4. Discussion

Ulcer is a major gastrointestinal disease that affects 10% of the world population [22]. Pyloric ligation is the most common method for induction of gastric lesions in rats. These lesions are induced *via* stimulation of histamine-2 receptors (H2R) leading to hypersecretion of hydrochloric acid (HCL) inside the stomach, and this increases gastric acidity and changes gastric pH [23]. Pylorus ligation induced hyperacidity causing autodigestion of the gastric mucosa and breakdown of the gastric mucosal barrier which resulted as upper gastrointestinal damage including lesions, ulcers, and hemorrhage. This leads to accumulation of gastric acid and development of ulceration in the stomach. Histamine-2 receptor blockers are reported as the most common antiulcer drugs with effectiveness against the pyloric ligation model [24]. The agents that decrease gastric acid secretion and increase mucus secretion are effective in preventing the ulcers induced by this method like ranitidine, acting as an antiulcer agent by an antisecretory mechanism *via* inhibition of gastric secretion. The effective antiulcer agents are attributed to their antisecretory and antilesion actions as the main initiator of ulcer formation is overproduction of gastric acid that causes erosion of the gastric mucosa and damages the gastric protective barrier [25]. Several studies were conducted by using natural extracts or oils for controlling gastric ulcers induced by different experimental methods [25].

In this study, we used new, natural, safe, inexpensive, and available extracts and oils to be tested and evaluate their antiulcerogenic activity such as *Aloe perryi* and date palm extracts in addition to yellow oil and red oil and also to explore their protective activities against gastric ulcer induced by pyloric ligation in rats and compare their action with the standard known antiulcer drug (H2 blocker such as ranitidine). *A. perryi* is a traditional herb with wide use in folklore medicine due to its safety and biological effectiveness [26, 27]. The *A. perryi* extract has many pharmacological activities. Recent study showed that the *A. perryi* extract has anti-inflammatory action and cytotoxic activities [28]. Moreover, another *in vivo* study showed its antidiabetic action due to hypoglycemic and insulin-releasing effects and hepatic antioxidant potentials in STZ-induced diabetic rats [29] and alloxan-induced diabetic rats [30]. Also, recent *in vitro* study showed antidiabetic and antioxidant activities of Aloe species [31]. *A. perryi* flower extracts showed *in vitro* antiproliferative and anticancer activities in the liver, lung, colon, breast, prostate, and epithelial human cell lines [12]. In this study, we used *A. perryi* leaf and flower extracts to be tested in another pharmacological action in the gastric ulcer model induced by the pyloric ligation method and to investigate gastroprotective effects of the two extracts against ulcer induction and progression. Chemically, the *A. perryi* flower extract possesses various pharmacologically important compounds such as essential oils, alkaloids, amino acids, anthraquinone glycosides, glycoproteins, vitamins, minerals, and lectins [12]. On the other hand, the *A. perryi* leaf extract contains many classes of bioactive compounds including chromones, flavonoids, anthraquinones, anthrones, amino acids, lipids, carbohydrates, vitamins, and minerals [28]. Also, we used date seed oil which contains many bioactive ingredients with variant biological activities. The date seed is mainly composed of dietary fiber, protein, carbohydrates, and minerals (potassium, magnesium, calcium, phosphorus, sodium, and iron). Such substances perform several functions from a biological point of view, such as antioxidant, antibacterial, and antiviral activities. Date seeds are also a good source of oil (5 to 13%), which is rich in phenolic compounds, tocopherols, and phytosterols [3, 6–9]. Date seed oil has been studied by other authors, and its composition of vitamins, minerals, and fatty acids makes it valuable for food formulations [9, 10]. The literature data confirm that date seed oil is an interesting source of important nutrients that have a very positive effect on human health [32].

Our results showed that pyloric ligation for 6 hours led to marked significant increases in total and free acidity, ulcer index, and hyperacidity of gastric content and decreased pH to being acidic, indicating the severity of this induction model of gastric ulcer. Moreover, histopathological study was performed that showed in macroscopic evaluation of gastric ulcer a deeply formed ulcer in the pyloric ligation method. The abovementioned changes indicated gastric ulcer formation by the pyloric ligation technique, and these observations were in accordance with previous studies' results [33, 34].

On the other hand, pretreatment with *A. perryi* and date palm extracts in addition to yellow and red oils for 1 hour before pyloric ligation has a protective effect against gastric ulcer progression which is confirmed by significant reduction of hyperacidity, total and free acidity, and ulcer index. Macroscopic evaluation of gastric ulcer showed normalization of the gastric mucosa without red spots, lesions, or perforations. These results showed the promising gastroprotective effects of *A. perryi* and date palm extracts in addition to yellow oil and red oil against the pyloric ligation ulcer model. These agents can be involved in gastric ulcer management.

## 5. Conclusion

Collectively, our findings demonstrated novel antiulcer activities of *Aloe perryi* and date palm extracts in addition to yellow oil and red oil in the pyloric ligation-induced gastric ulcer model as a result of antisecretory and mucosal strengthening properties. This is a preliminary study that may be a promising strategy to ameliorate the gastric ulcer associated with pyloric ligation, but further investigations are required to fully understand the action mechanisms of the extracts (Figure 6).

## Figures and Tables

**Figure 1:** Effect of the *A. perryi* leaf extract (APLE) and ranitidine on the percentage of ulcer inhibition in the pylorus ligation-induced ulcer model in the experimental rat model. APLE: rats received the *Aloe perryi* leaf extract in a dose level (250 and 500 mg/kg) (p.o.); ranitidine: rats received ranitidine which is dissolved in distilled water and given in a dose level (50 mg/kg) (p.o.) and served as a standard drug. *n* = 6/group.

**Figure 2:** Effect of the *A. perryi* flower extract (APFE) and ranitidine on the percentage of ulcer inhibition in the pylorus ligation-induced ulcer model in the experimental rat model. APFE: rats received the *Aloe perryi* flower extract in a dose level (250 and 500 mg/kg) (p.o.); ranitidine: rats received ranitidine which is dissolved in distilled water and given in a dose level (50 mg/kg) (p.o.) and served as a standard drug. *n* = 6/group.

**Figure 3:** Effect of the date palm seed extract (DPSE) and ranitidine on the percentage of ulcer inhibition in the pylorus ligation-induced ulcer model in the experimental rat model. DPSE: rats received the date palm seed extract in a dose level (250 and 500 mg/kg) (p.o.); ranitidine: rats received ranitidine which is dissolved in distilled water and given in a dose level (50 mg/kg) (p.o.) and served as a standard drug. *n* = 6/group.

**Figure 4:** Effect of oily samples of the date palm seed extract (DPSE) and ranitidine on the percentage of ulcer inhibition in the pylorus ligation-induced ulcer model in the experimental rat model. Yellow oil group: rats received date yellow oil in a dose level (250 and 500 mg/kg) (p.o.); red oil group: rats received date red oil in a dose level (250 and 500 mg/kg) (p.o.); ranitidine: rats received ranitidine which is dissolved in distilled water and given in a dose level (50 mg/kg) (p.o.) and served as a standard drug. *n* = 6/group.

**Figure 5:** Representative photomicrographs showing H&E-stained rat gastric sections. H&E-stained gastric sections revealed normal mucosal parts (arrowhead) followed by denuded part and remnant glands (thick arrow) without mucosal cells covered, congested blood vessels (thin arrow), and huge submucosal edema with lymphocytic infiltration and inflammatory aggregates (stars) (×100 magnification) (a). High magnification of the ulcerative surface with disruption and complete losses of all mucosal covered epithelium (gastric pits) and still low parts of the glandular layer which mixed with erythrocytes and individual inflammatory cells and/or destructed necrotic cells and congested deep blood vessels (arrow) (400x magnification in the control group) (b, c). Representative of the restoration of the mucosal structure (thick arrow) with still denuded and inflammatory cells individually between gastric glands (thin arrow) (100x magnification: amelioration findings in each APLE 250 mg/kg and DSPE 250 mg/kg group) (d). Representative of the restoration of mucosal surface structure with still minute ulceration surface (arrowhead) with mucosal necrosis and inflammatory cell aggregations (star) beside engorged blood vessels (thin arrow) (100x magnification: amelioration findings in each red oil DPSE 250 mg/kg, yellow oil DPSE, DSPE 500 mg/kg, APFE 500 mg/kg, and APLE 500 mg/kg) (f). Remodeling of all gastric structure layers with prominent normal gastric mucosa (100x magnification: amelioration findings in each red oil DPSE 500 mg/kg, ranitidine, and APFE 500 mg/kg group) (e).

**Figure 6:** Schematic diagram illustrating antiulcer activities of *Aloe perryi* and date palm extracts in addition to yellow oil and red oil in the pyloric ligation-induced gastric ulcer model.

**Table 1:** The ulcer protective effect of the *A. perryi* leaf extract (APLE) and ranitidine on the pylorus ligation-induced ulcer model in the experimental rat model.

Treatment	Dose	Parameters				
		Gastric volume (ml)	pH	Total acidity (mEq/l)	Free acidity (mEq/l)	Ulcer index
Control	1 ml/kg	8.47 ± 0.15	3.21 ± 0.13	120.83 ± 2.20	94.32 ± 0.31	3.58 ± 0.09
APLE	250 mg/kg	4.38 ± 0.11	4.47 ± 0.17^∗^	76.33 ± 1.17^∗^	65.67 ± 1.20^∗^	2.15 ± 0.05^∗^
	500 mg/kg	3.40 ± 0.07^a^	5.12 ± 0.11^∗^	66.83 ± 1.58^∗^	43.83 ± 1.22^∗^	1.34 ± 0.14^
Ranitidine	50 mg/kg	4.25 ± 0.21^∗^	5.35 ± 0.15^∗^	37.0 ± 0.17^∗^	17.0 ± 0.24^∗^	1.00 ± 0.03^∗^

Control: rats received only distilled water; APLE: rats received the *Aloe perryi* leaf extract in a dose level (250 and 500 mg/kg) (p.o.); ranitidine: rats received ranitidine which is dissolved in distilled water and given in a dose level (50 mg/kg) (p.o.) and served as a standard drug. *n* = 6/group. Values are expressed as mean ± SEM (*n* = 6). ^∗^*P* value is <0.001, ^a^*P* value is <0.01, and ^*P* value is <0.05 versus control.

**Table 2:** The ulcer protective effect of the *A. perryi* flower extract (APFE) on the pylorus ligation-induced ulcer model.

Treatment	Dose	Parameters				
		Gastric volume (ml)	pH	Total acidity (mEq/l)	Free acidity (mEq/l)	Ulcer index
Control	1 ml/kg	8.47 ± 0.15	3.21 ± 0.13	120.83 ± 2.20	94.32 ± 0.31	3.58 ± 0.09
APFE	250 mg/kg	3.62 ± 0.21^	5.52 ± 0.11^∗^	93.17 ± 1.30^∗^	84.00 ± 1.18^∗^	1.69 ± 0.03^∗^
	500 mg/kg	2.32 ± 0.12^∗^	6.73 ± 0.12^∗^	65.33 ± 1.38^∗^	48.67 ± 2.59^∗^	1.01 ± 0.03
Ranitidine	50 mg/kg	4.25 ± 0.21^∗^	5.35 ± 0.15^∗^	37.0 ± 0.17^∗^	17.0 ± 0.24^∗^	1.00 ± 0.03^∗^

Control: rats received only distilled water; APFE: rats received the *Aloe perryi* flower extract in a dose level (250 and 500 mg/kg) (p.o.); ranitidine: rats received ranitidine which is dissolved in distilled water and given in a dose level (50 mg/kg) (p.o.) and served as a standard drug. *n* = 6/group. Values are expressed as mean ± SEM (*n* = 6). ^∗^*P* value is <0.001 and ^*P* value is <0.05 versus control.

**Table 3:** The ulcer protective effect of the date palm seed extract (DPSE) on the pylorus ligation-induced ulcer model in the experimental rat model.

Treatment	Dose	Parameters				
		Gastric volume (ml)	pH	Total acidity (mEq/l)	Free acidity (mEq/l)	Ulcer index
Control	1 ml/kg	8.47 ± 0.15	3.21 ± 0.13	120.83 ± 2.20	94.32 ± 0.31	3.58 ± 0.09
DPSE	250 mg/kg	6.33 ± 0.15^∗^	2.7 ± 0.08	84.00 ± 1.34^∗^	74.33 ± 1.73^∗^	1.90 ± 0.06^∗^
	500 mg/kg	5.40 ± 0.10^∗^	3.4 ± 0.14	75.67 ± 1.38^∗^	56.67 ± 2.51^∗^	1.48 ± 0.10^∗^
Ranitidine	50 mg/kg	4.25 ± 0.21^∗^	5.35 ± 0.15^∗^	37.0 ± 0.17^∗^	17.0 ± 0.24^∗^	1.00 ± 0.03^∗^

Control: rats received only distilled water; DPSE: rats received the date palm seed extract in a dose level (250 and 500 mg/kg) (p.o.); ranitidine: rats received ranitidine which is dissolved in distilled water and given in a dose level (50 mg/kg) (p.o.) and served as a standard drug. *n* = 6/group. Values are expressed as mean ± SEM (*n* = 6). ^∗^*P* value is <0.001 versus control.

**Table 4:** The ulcer protective effect of oily samples of the date palm seed extract on the pylorus ligation-induced ulcer model in the experimental rat model.

Treatment	Dose	Parameters					
		Gastric volume (ml)	Total acidity (mEq/l)	pH	Free acidity (mEq/l)	Ulcer index	% of ulcer inhibition
Control	1 ml/kg	8.47 ± 0.15	120.83 ± 2.20	3.21 ± 0.13	94.32 ± 0.31	3.58 ± 0.09	—
Yellow oil	250 mg/kg	2.55 ± 0.11^∗^	66.50 ± 1.18^∗^	1.8 ± 0.05^∗^	54.50 ± 0.62^∗^	2.43 ± 0.05^∗^	32.1%
	500 mg/kg	2.38 ± 0.12^∗^	45.67 ± 1.41^∗^	2.2 ± 0.7^∗^	33.00 ± 0.82^∗^	1.61 ± 0.12^∗^	55.0%
Red oil	250 mg/kg	2.30 ± 0.14^∗^	76.33 ± 2.03^∗^	3.8 ± 0.06^∗^	58.83 ± 1.01^∗^	1.36 ± 0.06^a^	62.0%
	500 mg/kg	1.60 ± 0.11^∗^	56.50 ± 1.78^∗^	4.8 ± 0.07^∗^	36.00 ± 1.46^∗^	0.62 ± 0.05^a^	82.7%
Ranitidine	50 mg/kg	4.25 ± 0.21^∗^	37.0 ± 0.17^∗^	5.35 ± 0.15^∗^	17.0 ± 0.24^∗^	1.00 ± 0.03^∗^	72.1%

Control: rats received only distilled water; DPSE: rats received the date palm seed extract in a dose level (250 and 500 mg/kg) (p.o.); ranitidine: rats received ranitidine which is dissolved in distilled water and given in a dose level (50 mg/kg) (p.o.) and served as a standard drug. *n* = 6/group. Values are expressed as mean ± SEM (*n* = 6). ^a^*P* value is <0.01 and ^∗^*P* value is <0.001 versus control.

**Table 5:** Gross alteration scores for the gastric ulcer in control and treatment groups depending on mucosal color, hemorrhagic streaks, and deep or surface ulcer and perforation.

Findings	Control	Ranitidine	APLE		APFE		DPSE		Yellow oil		Red oil	
			250	500	250	500	250	500	250	500	250	500
Normal color	0	3	0	0	0	3	0	1	0	0	1	3
Red color	3	1	1	3	1	1	0	3	0	3	2	1
Hemorrhagic streak	3	0	2	3	3	0	3	2	3	2	1	0
Superficial ulcer	0	0	1	1	1	0	2	3		3	1	0
Deep ulcer	3	0	1	2	2	0	2	2	3	2	1	0
Perforation formation	0	0	0	0	0	0	0	0	0	0	0	0

Control: rats received only distilled water; APLE: rats received the *Aloe perryi* leaf extract in a dose level (500 mg/kg) (p.o.); ranitidine: rats received ranitidine which is dissolved in distilled water and given in a dose level (50 mg/kg) (p.o.) and served as a standard drug; APFE: rats received the *Aloe perryi* flower extract in a dose level (500 mg/kg) (p.o.); DPSE: rats received the date palm seed extract in a dose level (500 mg/kg) (p.o.); yellow oil group: rats received date yellow oil in a dose level (500 mg/kg) (p.o.); red oil group: rats received date red oil in a dose level (500 mg/kg) (p.o.). Gross severity scores: 0 = no changes, 1 = mild or focal, 2 = mild to moderate, and 3 = severe.

**Table 6:** Histological lesion scores for gastric alterations depending on loss of the mucosal and glandular layers, edema, and congested blood vessels with control and treatment doses and types.

Lesion	Control	Ranitidine	APLE		APFE		DPSE		Yellow oil		Red oil	
			250	500	250	500	250	500	250	500	250	500
Denudation of the mucosal parts	3	1	3	2	0.5	2	3	2	3	2	2	0
Congested blood vessels	3	0	3	1	1	1	3	1	3	1	1	0
Inflammatory cell infiltrations	3	0	2	1	2	1	2	1	2	1	1	0
Loss of the mucosal and glandular layers	3	0.5	3	2	1	2	3	2	3	2	2	0
Mucosal and/or submucosal edema	3	1	3	2	2	2	3	1	2	2	2	0
Regenerated tissues	0	2	1	2	1	2	1	1	0	1	1	3
Return to nearly normal feature	0	2	0	0	0	0	0	0	0	0	0	3

Control: rats received only distilled water; APLE: rats received the *Aloe perryi* leaf extract in a dose level (500 mg/kg) (p.o.); ranitidine: rats received ranitidine which is dissolved in distilled water and given in a dose level (50 mg/kg) (p.o.) and served as a standard drug; APFE: rats received the *Aloe perryi* flower extract in a dose level (500 mg/kg) (p.o.); DPSE: rats received the date palm seed extract in a dose level (500 mg/kg) (p.o.); yellow oil group: rats received date yellow oil in a dose level (500 mg/kg) (p.o.); red oil group: rats received date red oil in a dose level (500 mg/kg) (p.o.). The lesion scores: 0 = normal appearance; 0.5 = mild changes; 1 = moderate changes; 1.5 = severe changes; 2 = over severity; and 3 = diffused.

## Data Availability

All current results of this work are available with the corresponding author and can be provided upon reasonable request.
